# Microbiological Indoor and Outdoor Air Quality in Chicken Fattening Houses

**DOI:** 10.1155/2023/3512328

**Published:** 2023-05-29

**Authors:** Qadreyah A. Almatawah, Hanan S. Al-Khalaifah, Ahmad S. Aldameer, Abdulmohsen K. Ali, Ahmed H. Benhaji, Julie S. Varghese

**Affiliations:** Environment & Life Sciences Research Center, Kuwait Institute for Scientific Research, P.O. Box 24885, Safat 13109, Kuwait

## Abstract

This study was conducted at one of the largest poultry companies in Kuwait during November and December 2019 to evaluate the microbiological threats of *Escherichia coli* (APEC), *Salmonella* spp., and *Aspergillus fumigatus* to chickens in fattening houses by counting and identifying the microorganisms by culturing and pyrosequencing analysis. During the fattening cycle, the temperature and humidity ranged between 23.6°C and 29°C and 64.1% and 87.1%, respectively. The total bacterial population and *Aspergillus fumigatus* measured in the indoor and outdoor air exhibited a linear relationship during the fattening cycle. The total bacterial and *Aspergillus* concentrations determined during the cycle ranged between 150 and 2000 CFU/m^3^ and 0 and 1000 CFU/m^3^, respectively. *E. coli* and *Salmonella* spp. concentrations determined during the cycle ranged between 1 and 220 CFU/m^3^ and 4 and 110 CFU/m^3^, respectively. Pyrosequencing analysis of the air inside the houses at the end of the cycle revealed extensive biodiversity in the microorganisms, detecting 32 bacterial genera and 14 species. The identified species belonging to the genera *Corynebacterium*, *Haemophilus*, *Streptococcus*, *Veillonella*, and *Aspergillus* were identified as potentially affecting human and broiler health. The emission of potentially pathogenic bacteria to the outdoor environment from chicken housing can pose a considerable risk to human health and environmental microbial pollution. This study could guide the development of integrated control devices for monitoring microbes in broiler production facilities during chicken collection for transport to slaughterhouses.

## 1. Introduction

The accumulation of farming experience and the development of intensive and large-scale livestock production have made researchers more aware of the significant role that microbial aerosols play in epidemic spread, particularly respiratory diseases caused by pathogenic microbes [1, 2]. In livestock and poultry, the major infectious diseases are transmitted through the air, causing great harm and losses to the livestock industry, even threatening human health and obstructing the improvement and development of animal farming production efficiency. In the 1970s, researchers initiated the study of bioaerosols released during livestock and poultry farming processes [3, 4]. Bioaerosols contain a complex mixture of chicken and human-derived dander, chicken feed, bedding, and viable and nonviable microbial populations [5]. Many factors, including livestock and poultry species, farming methods, farming seasons, and stages, have been shown to affect the community structure of microbial aerosols [6, 7].

In poultry broiler production, exposure to bioaerosols in houses depends on the bird growth stage, as feather dandruff and feces biomass sharply increase during the fattening period. Moreover, during the fattened bird collection for transportation to the slaughterhouse, catching birds and placing them into boxes generate many supplementary bioaerosols. These bioaerosols can be inhaled by forklift operators while loading crates of chickens into transport. Time-based information on the quantity and microbial composition of bioaerosols is necessary to understand the relationship between these factors and adverse health symptoms in workers and animals.

The most commonly used technique for assessing bioaerosol microbial content is culture-dependent methods. This technique generated data that provide a quantitative measure of culturable bacteria and a low-resolution assessment of bacterial diversity. Nevertheless, knowledge of microbial diversity is limited because the vast majority (90–99%) of naturally occurring microorganisms cannot be cultured using standard techniques [8, 9]. On the other hand, real-time quantitative polymerase chain reaction (Q-PCR) is a molecular technique widely used in research areas where reproducible and accurate bacterial quantification is needed. The technique offers an attractive alternative method for quantifying the total microbial load and assessing species-specific profiles.

A great variety of microbial air concentrations in poultry houses and their surroundings are reported in the literature. In broiler houses, the reported concentrations of airborne microorganisms include up to 168,000 CFU/m^3^ [10], up to 46,000 CFU/m^3^ [11], and up to 220,000 CFU/m^3^ [12]. Around poultry houses, the reported number of microorganisms in the air (up to 500 m away from poultry houses) ranged from 2,200 CFU/m^3^ [13] to 21,000,000 CFU/m^3^ [14]. The composition of microbial air pollutant species has been studied and analyzed in detail [11, 15, 16]. The primary source of microbial contamination in poultry houses is birds, followed by feed, litter, and droppings; however, microbial counts are decreased primarily by the efficiency of ventilation systems [14].

Worldwide, avian colibacillosis, salmonellosis, and aspergillosis are important microbial diseases in the poultry industry. These diseases establish a significant public health problem and represent a high cost in many countries. Therefore, having a microbial air pollution database of poultry houses will assist poultry researchers and the poultry industry in reducing and eliminating avian colibacillosis, salmonellosis, and mycotoxins from poultry flocks, thereby reducing the potential hazards to public health posed by these bacterial diseases. The current database of microbial air pollution in poultry houses in Kuwait is insufficient at present. Hence, it is essential to collect and build a microbial database for poultry house air in Kuwait for the benefit of controlling broiler and human diseases. This study aimed to monitor the status of two of the most important airborne pathogens (*Escherichia coli* (APEC) and *Salmonella* spp.) and *Aspergillus fumigatus* in Kuwait's poultry houses.

## 2. Materials and Methods

### 2.1. Poultry Farm Studied

The poultry farm selected in this study represents one of the largest poultry companies in Kuwait. This farm is situated 50 km from the state capital of Kuwait and is located in areas reserved for the poultry industry. The poultry farm consists of 12 × 97 m broiler houses, each of which houses 20,000 birds. The broiler houses were decontaminated with glutaraldehyde and embedded with wood shavings prior to each fattening cycle. The houses are ventilated using a tunnel ventilation system. The birds are kept there until they reach 28 days of age. The prevalence of *E. coli*, *Salmonella* spp. and *Aspergillus fumigatus* in the air was determined from three selected broiler houses that received one-day-old chicks (Cobb-500) from the hatchery.

### 2.2. Microbial Contamination Analysis

Bioaerosols were sampled by impaction and impingement prior to the placement of the chicks and during the grow-out period. The samples were collected weekly from areas containing ventilation fans in the three houses. Duplicate samples for *E. coli* and *Salmonella* were collected in 20.0 ml of pyrogen-free saline (0.09% NaCl) using an impinger operating at a flow rate of 12.5 L/min for 10 min. In the impaction method, samples were impacted onto XDL, MacConkey, and sorbitol MacConkey plates at a flow rate of 28.3 L/min for 10 min, using an impactor [17]. The impinger sample solutions were concentrated to 1 ml and stored at −20°C for DNA analysis. *Aspergillus fumigatus* was collected with the impact method using malt extract agar supplemented with chloramphenicol (0.5%) to inhibit bacterial growth. Field and shipping blanks were collected for quality control procedures [18]. All sampling devices were operated in the morning and were placed at 0.5 m and 1.5 m above the floor. Air temperature and humidity were recorded during the sampling using a Supco DSP990 digital psychrometer (Sealed Unit Parts Co., Inc., New Jersey, USA).

### 2.3. Microbial Detection and Characterization by the Standard Culture Method

Plates from the impaction procedure were incubated at 37°C for *E*. *coli* and *Salmonella* and at 30°C for *Aspergillus fumigatus*. Colonies were counted after 48 h of incubation for bacteria and after 5 days for molds; subsequently, the colony-forming units (CFUs) were determined. The concentration of microorganisms in colony-forming units per metric cube (CFUm^−3^) was computed based on the number of colonies counted on the plates (*N*) as described by the following equation [19, 20]:

(1) $$\begin{array}{c} Concentration\left({CFUm}^{-3}\right)=10^{3}\times \frac{N}{Q}\times t\text{,} \end{array}$$

where *Q* is the flow rate of the sampling pump (L min^−1^ and the sampling time is indicated by *t* (min)). Isolated colonies were further confirmed for *E. coli* and *Salmonella* spp. using biochemical confirmation (Biolog Gen III Omnilog®II Combo System). Antibiotic sensitivity for the isolated strain at different concentrations was performed using the standard paper disc diffusion method described by the NCCLS [21]. Identification of filamentous fungi was carried out by microscopic examination of the culture and the fungal material mounted in lactophenol blue stain.

### 2.4. Assessment of Microbial Diversity by Pyrosequencing Analysis

Whole community genomic DNA was extracted from 1 ml concentrate from a total of 12 air samples from the last week in the fattening cycle using the Water RNA/DNA Purification Kit (0.22 *μ*m, NGB-26400, Norgen Biotek Corp., Warburgstr, Hamburg, Germany), according to the protocol provided by the manufacturer. Each sample represents three samples from each of the three houses, which were pooled to create three pools of DNA. Extracted DNA (2 *μ*L) was checked for purity and concentration using an Invitrogen™ Qubit™ 3 Fluorometer (Thermo Fisher Scientific, San Francisco, CA, USA) and was run on a 0.8% agarose gel. DNA pyrosequencing was performed by Beijing Genomics Institute (BGI Shenzhen, China). In brief, the PCR mixtures (50 *μ*l) contained 30 ng of sample DNA, 25 *μ*l of NEB Phusion High-Fidelity PCR Master Mix (New England Biolabs, USA), and 4 *μ*l each of forward and reverse primer 16SV4 (515F-806R) [22]. The reaction was carried out in Veriti Thermal Cyclers (Applied Biosystems, Grand Island, NY) with an initial activation of the DNA polymerase at 98°C for 3 min, followed by 30 cycles at 98°C for 45 s, 55°C for 45 s, 72°C for 45 s, and a final extension step at 72°C for 7 min. The PCR products were visualized on a 1.8% agarose gel that was run at 150 V for 40 min and purified with Agencourt Ampure XP beads (Beckman Coulter, USA) to remove the nonspecific products. The final library was quantitated in two ways. First, the average molecule length was determined using an Agilent 2100 bioanalyzer instrument with Agilent DNA1000 Reagents (Agilent Technologies, USA), and the library was quantified by real-time quantitative PCR. Second, the library was quantified by a StepOne plus real-time PCR system (Applied Biosystem, USA) and EvaGreen Kit (Biotium, USA). High-throughput sequencing of the qualified libraries was conducted by using the Illumina MiSeq platform (Illumina, USA) and MiSeq Reagent Kit. Raw data were filtered to eliminate adapter pollution and low quality to obtain clean reads, and then, paired-end reads with overlap were merged into tags. The tags were clustered to operational taxonomic units (OTUs) at 97% sequence similarity. The reads were merged using the FLASH program (version 1.2.11) with a minimum overlap of 15 bp, ≤0.1 mismatches yielding, and an average contig length of 252–291 bp. OTU representative sequences were taxonomically classified using Ribosomal Database Project (RDP) Classifier v.2.2 which was trained on the database Greengene_2013_5_99, using 0.6 confidence values as a cutoff. Finally, alpha diversity, beta diversity, and the screening of different species were analyzed on the basis of OTUs and taxonomic ranks.

### 2.5. Statistical Analyses

The temperature and relative humidity values and bacterial count in the air were analyzed using Microsoft Excel 2016 MSO and SPSS software for Windows, version 28.0, including descriptive statistical analysis and statistical significance at the 5% level (*P* < 0.05). Analysis of variance (ANOVA) was performed on indoor and outdoor concentrations of bacteria and fungi using week as the main parameter. To study the relationship between indoor and outdoor air microbial concentrations during the fattening cycle, Pearson's correlation coefficient was used.

## 3. Result

### 3.1. Microbial Contamination Analysis

The studies were carried out in the autumn of 2019, when the atmospheric air temperature ranged between 21.6°C and 32.2°C, and the inside temperature in the poultry houses varied from 23.6°C to 29°C. Relative air humidity ranged between 64.1% and 87.1% indoors and between 25% and 71% outdoors. Microbial contamination analysis data showed an increase in the total bacterial count inside and outside the houses' air during the fattening process (Figure 1). The maximum count was reached in the second week of the process, and then, the count decreased in the fourth week. Figures 2–4 clearly show the percentage increase in the microorganisms under study (*E. coli*, *Salmonella*, and *Aspergillus*) compared with other bacterial counts inside and outside the houses during the autumn fattening process. Figures 5–7 demonstrate the increase in *E. coli*, *Salmonella*, and *Aspergillus* counts during the fattening process. During the process, indoor and outdoor air showed an increase in *E. coli*, *Salmonella*, and *Aspergillus* counts, with the maximum count in the second week at 0.5 m. Only *E. coli* showed a maximum count in the third week of the process at 1.5 m, inside and outside the air. In addition, the first week had the highest number of *Salmonella* in the outdoor air.

At the 1.5 m detection level, the total bacterial concentration in the fattening houses during the process ranged from 150 ± 160 to 2000 ± 600 CFU/m^3^ (Table 1), which was linearly related to the outdoor air during the fattening cycle (Figure 8). The highest concentration was detected in the second week of the process. The concentrations of *E. coli, Salmonella*, and *Aspergillus* during the process ranged from 1 ± 2 to 220 ± 250 CFU/m^3^, 4 to 110 ± 43 CFU/m^3^, and 0 to 610 ± 160 CFU/m^3^, respectively, with the highest concentration in the second week of the process (Table 1). There was a strong positive and significant correlation between the total number of bacteria and *Aspergillus* in the air inside and outside the house at 1.5 m (*r* = 0.995 and 0.996, respectively; *P* < 0.001) (Table 2). The ANOVA test performed on total raw data revealed significant differences in the total bacterial and *Aspergillus* indoor contamination related to the week (Table 3). Inside the houses, at the 0.5 m detection level, the relationship between microbial concentration and the fattening cycle week was insignificant only for total bacterial count and *Salmonella* (*P* > 0.05). However, at the 1.5 m detection level, the relationship was insignificant only for *E. coli*. Additionally, outside the houses, at the 1.5 m detection level, the relationship was insignificant only for *E. coli*.

The indoor/outdoor ratio (I/O; Table 1) was calculated using the indoor and outdoor microbial counts obtained during the fattening process sampling at 1.5 m. At 1.5 m, the human birthing level and I/O ratios showed that maximum counts for the total bacteria in autumn were lower indoors than outdoors during the fatting process (I/O values close to one or more bacterial counts indicated higher bacterial contamination inside the building than outside). Furthermore, I/O ratios showed that maximum counts for *E. coli*, *Salmonella*, and *Aspergillus* during autumn were lower indoors than outdoors during the fattening process. All the target houses had indoor sources of airborne bacteria, which contaminated the indoor air. The outdoor air contamination level was assessed according to Polish Norm standards (Table 4). In the first week of the chicken fattening cycle at 1.5 m, the total bacterial counts were 2000 CFU/m^3^, which means that the houses were polluted with a medium extent of pollution. At 0.5 m, the counts from the first week to the third week were high: 1230 CFU/m^3^, 1438 CFU/m^3^, and 1131 CFU/m^3^, respectively. Biochemical analysis of the isolated strains in the third week of the fattening cycle confirmed the presence of *E. coli* and *Salmonella* species (*S. enterica* and *S. subterranean*). However, avian pathogenic *E. coli* (APEC) was not detected. *Aspergillus fumigatus* was detected by microscopic methods.

### 3.2. Microbial Diversity in Chicken Fattening Houses

The analysis of bacterial diversity at the genus and species levels at the end of the fattening cycle-pooled DNA is shown in Figures 9 and 10, respectively. The tag number of each taxonomic rank (genus, species) in different samples was summarized in a profiling histogram. Figures 9 and 10 show the taxonomic composition distribution histograms of indoor and outdoor samples at the genus and species levels, respectively. The species with less than 0.5% abundance in all samples were classified into “others” in other ranks.

In the indoor samples, the dominant genus identified was *Corynebacterium* (25.1%), followed by *Streptococcus* (15.2%), *Staphylococcus* (9.7%), *Haemophilus* (7.3%), *Agrobacterium* (5.5%), *Actinomyces* (2.9%), *Burkholderia* (2.3%), *Anaerococcus* (1.9%), *Alloiococcus* (1.6%), *Veillonella* (1.5%), *Achromobacter* (1.4%), and *Lactococcus* (1.2%). In the outdoor samples, the dominant genus was *Agrobacterium* (38.5%) followed by *Burkholderia* (25.1%), *Corynebacterium* (10%), *Staphylococcus* (7%), *Achromobacter* (2.9%), and *Streptococcus* (1.3%) (Figure 9). Both indoor and outdoor samples were mainly contaminated with bacteria belonging to the genera *Streptococcus* and *Staphylococcus*. The *Streptococcus* genus was the predominant genus inside the houses.

The species analysis revealed that in the autumn indoor samples, the dominant species identified were *Streptococcus infantis* (13.7%) followed by *Haemophilus parainfluenzae* (7.3%), *Corynebacterium kroppenstedtii* (3.4%), *Veillonella parvula* (1.5%), and *Streptococcus anginosus* (1.3%). In the outdoor samples, the dominant genus was *Corynebacterium kroppenstedtii* (2.3%), followed by *Streptococcus infantis* (0.9%), *Streptococcus anginosus* (0.3%), *Haemophilus parainfluenzae* (0.2%), and *Veillonella parvula* (0.2%) (Figure 10). *Streptococcus infantis* was the predominant species inside the houses.

## 4. Discussion

Counting and monitoring aerial microorganisms inside and outside poultry farms are essential for evaluating the impact of poultry houses on environmental microbiological pollution [24]. Collecting temporal information on the quantity and composition of bioaerosols is necessary to better understand the relationship between these factors and adverse health symptoms in workers and animals. The numbers and types of airborne bacteria are useful indicators for assessing the adverse effects of human exposure to these emissions [25]. This human health risk assessment is used to assess health hazards associated with exposure to airborne bacteria and fungi [26]. The concentrations and emissions of pathogenic bacteria and fungi in the air depend on the health of the chickens when they are raised in the poultry house.

In this study, the total bacterial population measured in the indoor air and outdoors exhibited a linear relationship during the fattening cycle, with an *R*^2^ of 0.8349. Pyrosequencing analysis of the indoor and outdoor air in chicken fattening houses revealed a large diversity of bacteria in indoor and outdoor air. During the last week of the fattening cycle, a comprehensive DNA analysis was performed on air samples collected from (inside) and (surrounding) poultry houses to identify pathogenic bacteria present during chicken collection for transport to slaughterhouses. The analysis of indoor air samples demonstrated that Gram-positive bacterial species, such as *C. kroppenstedtii*, *S. anginosus*, and *S. infantis,* and Gram-negative bacterial species, such as *H. parainfluenzae* and *Veillonella parvula,* are highly abundant in poultry house air during autumn. *E. coli* was detected in less than 0.02%, whereas *Salmonella* spp. was not detected; however, *Salmonella* spp. was detected by culture methods in the third week of the process by biochemical analysis. The inability to detect *Salmonella* spp. is in agreement with a previous study [27] that found that *Salmonella* spp. prevalence in poultry farms is sporadic [28]. The detected bacterial species belonging to the genera *Corynebacterium*, *Haemophilus*, *Streptococcus*, and *Veillonella* were potentially harmful to humans [29–39]. Moreover, the detected *Aspergillus* species are also potentially harmful to humans and broilers [40–42]. These pathogenic bacteria and fungi were present in a higher percentage inside the house's air than in the air outside, reflecting the emission of these microorganisms from the inside air. Although the calculated 1/O reflected no pollution, the pyrosequencing analysis of the indoor and outdoor air showed the emission of harmful bacteria to the outdoor environment. The discharge of potentially pathogenic bacteria from chicken housing to the outdoor environment can pose a considerable health risk to humans and environmental contamination.

## 5. Conclusion

Poultry houses are a source of significant emissions of microbial pollutants into the atmospheric air. Large discharges of this potentially pathogenic microorganism into the outdoor environment via aerosols from poultry breeding facilities may pose a considerable risk to human health and environmental microbial contamination. To date, there are no reliable data on the relationship between indoor and outdoor microbial contamination in poultry houses in Kuwait. This study highlights that poultry houses have the potential to transmit diseases through airborne bioaerosols; therefore, corrective actions are needed to mitigate negative public health impacts. Consideration should be given to establishing an appropriate monitoring system to reduce the types and concentrations of bioaerosols in the air and to take measures to control microbial contamination in the air.

## Figures and Tables

**Figure 1:** CFU/m^3^ for total bacterial count during the 4-week autumn fattening cycle at 0.5 m and 1.5 m air above the floor inside the houses and at 1.5 m air outside the houses.

**Figure 2:** Percentage of microorganisms (CFU/m^3^) during the 4-week autumn fattening cycle at 0.5 m air above the floor inside the houses.

**Figure 3:** Percentage of microorganisms (CFU/m^3^) during the 4-week autumn fattening cycle at 1.5 m air above the floor inside the houses.

**Figure 4:** Percentage of microorganisms (CFU/m^3^) during the 4-week autumn fattening cycle at 1.5 m air above the floor outside the houses.

**Figure 5:** CFU/m^3^ for *E. coli*, *Salmonella*, and *Aspergillus* during the 4-week autumn fattening cycle at 0.5 m air above the floor inside the houses.

**Figure 6:** CFU/m^3^ for *E. coli*, *Salmonella*, and *Aspergillus* during the 4-week autumn fattening cycle at 1.5 m air above the floor inside the houses.

**Figure 7:** CFU/m^3^ for *E. coli*, *Salmonella*, and *Aspergillus* during the 4-week autumn fattening cycle at 1.5 m air above the floor outside the houses.

**Figure 8:** Correlation between microbial concentrations in the air samples at 1.5 m above the floor inside and outside the houses during the fattening cycle.

**Figure 9:** The taxonomic composition distribution in samples of genus level. (1) Autumn indoor sample. (2) Autumn outdoor sample.

**Figure 10:** The taxonomic composition distribution in the samples at species level. (1) Autumn indoor sample. (2) Autumn outdoor sample.

**Table 1:** Microorganisms mean CFU per cubic meter of air range during the four weeks fattening cycle inside and outside the houses and I/O for maximum counts.

Microorganisms	CFU/m^3^ range			I/O^*∗*^
	0.5 m (in)	1.5 m (in)	1.5 m (out)	
Total bacteria	400–1230	150–2000	230–2480	0.78
*E. coli*	2–300	1–220	0–230	0.97
*Salmonella* spp.	6–240	4–110	4–400	0.75
*Aspergillus fumigatus*	0–850	0–610	0–1000	0.61

^*∗*^I/O at 1.5 m detection level.

**Table 2:** Pearson's correlation coefficient (*r*) between microbial concentrations in indoor and outdoor air during the fattening cycle.

Microorganisms	Correlation detection location	Person correlation	*P* value
Total bacteria	0.5 m (in)–1.5 m (in)	0.712	0.178
	0.5 m (in)–1.5 m (out)	0.661	0.225
	1.5 m (in)–1.5 m (out)	0.995	<0.001

*E. coli*	0.5 m (in)–1.5 m (in)	0.039	0.950
	0.5 m (in)–1.5 m (out)	−0.246	0.691
	1.5 m (in)–1.5 m (out)	0.882	0.048

*Salmonella* spp.	0.5 m (in)–1.5 m (in)	0.856	0.064
	0.5 m (in)–1.5 m (out)	−0.088	0.888
	1.5 m (in)–1.5 m (out)	0.031	0.961

*Aspergillus fumigatus*	0.5 m (in)–1.5 m (in)	0.992	0.178
	0.5 m (in)–1.5 m (out)	0.997	0.225
	1.5 m (in)–1.5 m (out)	0.996	<0.001

**Table 3:** The analysis of variance on bacterial and *Aspergillus* counts with respect to week.

Microorganism	*P* value		
	0.5 m (in)	1.5 m (in)	1.5 m (out)
Total bacteria	0.06	<0.001	<0.001
*E. coli*	0.018	0.440	0.104
*Salmonella* spp.	0.472	0.004	<0.001
*Aspergillus fumigatus*	<0.001	<0.001	<0.001

**Table 4:** Polish Norms PN-89/Z-04111/02 and PN-89/Z-04111/03 (https://www.pkn.pl/) [23].

Polish Norm	Mesophilic bacteria	Staphylococci	Fungi
No pollution^*∗*^	<1000	0	3000–5000
Medium pollution^*∗∗*^	1000–3000	<25	5000–10000
Heavy pollution^*∗∗∗*^	>3000	>25	>10000

## Data Availability

The original contributions presented in the study are included within the article, and further inquiries can be directed to the corresponding author.
